# English Education Tutoring Teaching System Based on MOOC

**DOI:** 10.1155/2022/1563352

**Published:** 2022-05-27

**Authors:** Wang Mi

**Affiliations:** Zhejiang Industry and Trade Vocational College, Wenzhou, Zhejiang 325000, China

## Abstract

In the process of continuous reform and development of education and teaching, some traditional teaching modes are gradually eliminated, whereas new teaching modes are gradually recognized by teachers and students. These modes are widely used in education and teaching due to their overwhelming characteristics. Among these emerging teaching modes, massive open online course (MOOC) is a relatively advanced teaching mode with a better application effect. Quickly and accurately detecting the cheating behavior of MOOC learners is of great significance for maintaining the development of the MOOC platform and English education counseling. This paper studies a deep-learning-based hybrid model for MOOC cheating detection. The model greatly improves the detection performance of a single model by integrating CNN, a bidirectional gated recurrent unit, and an attention mechanism. The proposed model selects the English learning behavior data of a MOOC platform to verify the performance of the algorithm. Simulation results show that the proposed scheme can greatly help MOOC-based English education tutoring.

## 1. Introduction

With the ongoing growth of the Internet and information technology, a new sort of teaching mode with a modern nature has risen in recent years, that is, MOOC, which is defined as massive open online course. It relies heavily on advanced information technology and network platforms in order to carry out the necessary education and teaching tasks. Teaching concepts are mostly based on students' self-directed learning, with some direction and explanation provided by the teacher as a supplement [1–5]. Traditional knowledge installation is given more importance in the MOOC teaching approach, which emphasizes interaction and discussion between lecturers and students. Specifically, it is to carry out education and teaching activities in an equal relationship between teachers and students in order to better achieve the improvement of students' learning outcomes [6–8].

The most significant feature of MOOCs is the two-way flow of information as compared to the traditional teaching methods available in literature. It is due to the fact that in the MOOC teaching method, students can discuss the difficulties they have encountered in their own learning or the areas of the teaching that they do not understand [9, 10]. The problems or issues are conveyed to the teacher in the form of a message, and the teacher can understand the students' learning situation. Additionally, existing problems in the teaching through the feedback of the students allow not only for targeted guidance to be provided to some students but also for effective improvement and reform in the teaching content and teaching methods [11–13].

The properties of MOOCs are considerably different from those of traditional instructional approaches. In general, MOOCs are distinguished by the following characteristics: as a starting point, they exhibit qualities of openness during the learning process. An online open course (MOOC) differs from a regular classroom environment. Student learning is restricted by the constraints of time and place in traditional classroom settings. Students, on the other hand, can access the learning platform at any time and from any location when the MOOC teaching mode is in effect. Students' needs for autonomous learning can be met efficiently through interactive learning, which is possible as long as there is a network and appropriate equipment. Second, the substance of the lessons demonstrates features of variation. MOOCs are an information-based teaching method that relies on the Internet platform. As a result, the teaching content can be improved by drawing on a wealth of Internet-based educational resources, and students can also broaden their learning experiences by participating in MOOCs. Students should choose resources for learning that are reasonable for them based on their own preferences and learning needs. This is more favorable to the realization of students' individualized learning and can boost students' learning interest and efficiency [14–18].

In the online mode of instruction, there is a lack of necessary supervision, which results in the phenomena where learners achieve corresponding learning tasks by cheating, such as brushing courses, plagiarizing, or taking tests. In recent years, colleges and universities have begun to recognize MOOC credits as legitimate academic credits, making it critical to identify and prevent MOOC cheating habits [19–25].

When it comes to the cheating issue in MOOCs, there are two traditional remedies. One method is to utilize passive protection to prevent learners from cheating or to raise the difficulty of cheating by increasing the difficulty of cheating. Other options include employing active detection technology to identify cheating behavior and dealing with it in a timely manner in order to limit the prevalence of cheating [26, 27]. With regard to the first option, it is typically recommended that learners be prevented from engaging in some criminal activities throughout the online learning process by technical means. In order to prevent students from engaging in illegal activities such as page switching, answer copying, and mutual plagiarism, some illegal operations are disabled or blocked by means of the operating system kernel API calling technology, system message interception technology, callback technology, hook technology, registry access technology, and so on. In practice, however, this method of preventing cheating through technical means is frequently insufficient because the computer system is large and complex. Furthermore; because this hard-coded protection method is ineffective under the new cheating method, it is still necessary to employ detection technology. Cheating has been discovered [28–30].

Engineering applications for MOOC cheating behavior detection are typically carried out by combining manual detection and rule detection; however, this method not only consumes a large amount of manpower and material resources but also has drawbacks such as low detection efficiency and poor detection effect. Regarding academic research, several researchers have developed a cheating detection system based on mutual plagiarism that is based on data collected from candidates during online examinations. The CAMEO (copying answers using multiple accounts) method has been used by other researchers to design an algorithm to identify cheating learners. This method builds an IP-independent algorithm by evaluating the impact of learner, question, and submission characteristics on CAMEO. CAMEO learners are identified using a random forest classifier. In order to obtain the corresponding features, some researchers created some indicators and then used the K-means clustering algorithm to group them together in order to identify the use of these two cheating methods, which include sharing answers with one another and creating fake accounts in order to obtain correct answers. Both ways of cheating are taught to students [31–35].

In the course of the learning process, learners take a variety of learning action paths that differ from one another. Normal learners, for example, will view the learning video first, then do the tasks, and finally submit their answers. Abnormal learners may choose to practice exercises directly or concentrate on a specific time period for brushing, for example. In essence, the identification of cheating activity in MOOCs falls within the category of aberrant behavior detection problems.

The challenge of aberrant behavior detection is prevalent in a wide range of domains, including network intrusion detection, credit card fraud detection, defect detection, and household electricity detection, among others. Abnormal behavior detection algorithms can be divided into two categories, according to existing literature research. The first category includes traditional machine learning algorithms based on manual feature extraction, and the second category includes deep learning algorithms based on automated feature extraction. Traditional machine learning algorithms, on the other hand, rely far too heavily on human feature extraction, which is frequently insufficient, resulting in poor model performance and other issues. As a result, several researchers are attempting to apply deep-learning-based approaches for the detection of deviant behavior.

The studies mentioned above are all directed at a certain type of cheating, and after developing appropriate features, they employ statistical or machine learning methods to detect cheating in such situations. The ability to quickly and reliably detect the cheating behavior of MOOC learners is critical for the further growth of the MOOC platform as well as the provision of English language education guidance. For this reason, the research investigates a more general cheating detection model that is capable of solving numerous forms of cheating.

The rest of the paper is arranged as follows:

In Section 2, the significance and innovative ways of applying the MOOCs in English teaching is presented with a detailed discussion on it various subsection such as significance, value, and so on. In Section 3, a detailed analysis of the CNN-GRU-attention (CGA) for the MOOC cheating detection model is presented. Experimental observations are reported in Section 4 of the manuscript that is followed by the conclusion section.

## 2. The Significance and Innovative Ways of Applying MOOCs in English Teaching

### 2.1. Significance and Value

#### 2.1.1. Helping to Improve Students' Learning Enthusiasm and Autonomy

As a result of their inability to keep up with the pace of the instruction, some students with weak English foundations eventually lose confidence in their ability to learn English in the traditional English teaching mode. In English teaching, it is impossible to actively participate in the classroom and engage in effective independent learning. This will surely impede the smooth progression of the curriculum and the steady increase of students' English language ability. Although not perfect, the MOOC learning model efficiently tackles the problem of fixed traditional teaching content and form along with providing students with a greater number of options. Students can choose to study in a reasonable manner according to their current situation, regardless of whether they have a good or a weak foundation. Students' English ability can be continuously improved on an original basis through MOOC learning if they have access to appropriate resources and learning methodologies. Furthermore, students can communicate and interact effectively in the MOOC learning mode, allowing some students with weak foundations to solve problems in a timely manner by communicating and discussing with their classmates, which not only improves the students' learning ability but also helps them become better communicators and interactors. This method can also help students who have a weak foundation experience a sense of accomplishment in their learning, so increasing their excitement for and autonomy in their English study.

#### 2.1.2. Conducive to Cultivating Students' English Application Ability

Most of the purpose of education is to cultivate some generalized capabilities with great application abilities. As a result, in English teaching, the purpose is not only to transfer a great deal of English knowledge and grammar to students but also to place a strong emphasis on cultivating students' English proficiency. The capacity to apply English knowledge and grammar in a flexible manner in a real-world setting is demonstrated by students' ability to successfully perform English communication tasks. It is difficult to see the benefits of cultivating pupils' abilities in this area when English is taught in the usual manner. Despite the fact that pupils have a particularly strong command of English grammar and vocabulary, they are unable to attain greater results in practical application. Students can benefit from the MOOC teaching mode because they have access to more rich and diversified learning resources, and their horizons are broadened as a result. Furthermore, the MOOC teaching method provides students with an online oral communication platform, which allows them to communicate with other students who are also using the platform to converse. You can also immediately contact overseas pals in English if you want to conduct spoken communication and dialogue with them. The purpose of this process is not only to facilitate cross-border linguistic interchange but also to facilitate cross-border cultural exchange in order for students to gain more knowledge, enhance their knowledge, and also learn more about other cultures. It enables students to master the application of English information in a variety of contexts and environments, thereby significantly improving their English application skills.

#### 2.1.3. Conducive to Improving the Quality of English Teaching

In English teaching, the traditional teaching approach does not produce the best results because the students themselves have a weak foundation, and there are also significant discrepancies in the English education acquired by students from different geographical locations. Students brought about a great deal of hardship. Furthermore, both teaching content and teaching methods in traditional English teaching are relatively fixed and single, that is to say, a one-size-fits-all teaching method is adopted in traditional English teaching, which results in some students with stronger foundations being unable to communicate effectively in the language of instruction. Students with inadequate foundations will appear to be extremely tough to study if their foundations continue to strengthen.

### 2.2. Innovative Ways

#### 2.2.1. Constructing a Distinctive English Curriculum System in the Context of MOOCs

To build a more distinctive English curriculum system for students, create distinctive English teaching courses, and prioritize cultivating students' English application ability as one of the most important goals of teaching in the context of MOOCs, English teaching should combine students' learning needs and MOOC teaching concepts. One is to significantly improve students' ability to use English in various situations. It is possible to improve the sharing of educational materials, better integrate students' learning needs, and create a better English learning environment for students by developing a distinctive English teaching system. When developing the English characteristic teaching system, the curriculum system should be separated into sections based on the demands of the students' growth. This will allow the English teaching to be more targeted and the development of students' English ability to be more effective.

For example, in MOOC-based curriculum development system, teachers are able to assign modules from three aspects, namely basic modules, professional-English modules, and comprehensive quality modules. These modules correspond to the knowledge objectives, ability objectives, and quality objectives. The MOOC design has the potential to provide students with a wealth of educational resources. Teachers should consider the development of professional talents as the primary goal of their English MOOCs for a certain major when planning their English MOOCs. When creating MOOCs, mix English courses with professional courses, boost professional vocabulary, and enrich students' English professional knowledge by including them in the production, depending on the pupils' ability. Specifically, in terms of development, teachers can use MOOCs to design different listening, speaking, reading, writing, and translation content for students and use the advantages of courses to conduct intensive training for students while at the same time guiding students to study independently, emphasizing the benefits of MOOCs, and realizing the integration of MOOCs into teaching. In-depth integration is required. In addition, professors could use MOOCs to develop hands-on training courses for their students. For example, according to the tour guide profession, simulating on-site learning scenarios can help students integrate their newly acquired knowledge into the real world of work, create a classroom environment conducive to active learning and application, and improve the effectiveness of their practical training. Improve pupils' ability to communicate effectively in English as a professional.

As a matter of course, teachers should adhere to the construction principle of “student-centeredness” in the process of developing the English unique teaching system. Students are the primary constituents of the MOOC as well as the primary recipients of education and training. The use of MOOCs and the development of a teaching system are also intended to help students learn more effectively. Students will be better able to carry out their studies and serve. Because of this, when developing the system, it is vital to take into consideration the actual circumstances of pupils. Students and students, for example, have a significant disparity in terms of English foundation when compared to one another. The curriculum system can be designed for high and middle schools based on the lower three levels of teaching content and learning starting point, allowing the course content to be more humanized and students to choose their own learning content and starting point during the course construction process.

#### 2.2.2. Make Full Use of MOOC Resources to Enrich the Content of English Teaching in the Context of MOOCs

The effectiveness of English language instruction has substantially improved in the setting of MOOCs. It is due to the implementation of the MOOC platform that encourages students to take more responsibility for their own learning. Despite the fact that MOOCs can help students study more effectively on their own and create better learning environments for them, traditional classroom instruction is still necessary. In order to promote the double come of the core language class of the bureau, the teaching substance of the FTV lecture has been significantly increased in order to provide students with a more positive classroom learning experience. Even in the setting of massive open online courses (MOOCs), English classroom instruction continues to perform an essential and indispensable function. It is possible to think of classroom instruction as a standardized guide for students' learning. Students can achieve greater results by conducting MOOCs on their own time, rather than relying on traditional classroom instruction. The educational resources contained in MOOCs are extremely rich and diversified, and English teachers should take advantage of this to effectively expand the teaching content in accordance with the demands of their students in the traditional classroom.

#### 2.2.3. Constructing a Flipped Classroom to Innovate Higher Vocational English Teaching Methods in the Context of MOOCs

It is necessary to reform and reinvent English education in the context of massive open online courses (MOOCs) in order to provide customized instruction. Aside from being convenient, MOOCs are also beneficial for the optimization and development of focused English instruction. English teachers can implement this teaching reform by establishing a flipped classroom, in which teachers allow students to conduct targeted autonomous learning after class in accordance with the teaching design established before class, and students can learn through MOOCs (massive open online courses). Create settings that allow teachers to demonstrate to students their autonomous learning successes after class and to offer students a positive environment for oral English conversation. Teachers should make full use of MOOC teaching resources in the reformation of this teaching technique so that students may learn freely and can answer their own misunderstandings during the exchange and discussion in class, allowing them to retain the knowledge they have gained. Enhance their abilities to apply in English and make more effective applications.

Teachers in spoken English classes, for example, may assign MOOC resources to students based on various scenarios, such as those encountered at airports and customs, hotels and restaurants, asking for directions, shopping, claiming tax refunds, and seeing the doctor. Teaching guidance suggests that the teachers first concentrate on teaching for 20 minutes a day, then use the MOOC to explain to the students, grabbing their attention, requiring the students to gain a comprehensive understanding of the topic in a short period of time, and laying a solid foundation for the student's oral English. Basic. The pupils are then forced to pronounce “punch-in” on a daily basis, which is done through a WeChat group. The teacher examines the students' learning environment, corrects the students' oral pronunciation errors as soon as they occur, and guides the students' oral pronunciation. In the after-class guidance, the teacher delivers the pronunciation video to the students once more to guide them through the process. Read the passage and highlight the areas where mistakes are likely to occur to encourage students to pay attention to the pronunciation. Finally, the teacher packs and uploads the video, and students are required to play it again independently every day, summarize and reflect on the knowledge points that are confusing in the topic, complete the assignment, and post it to the platform to demonstrate their understanding. Students not only can benefit from centralized learning through MOOCs but also can benefit from having their own individual learning areas. It can be shown that the English flipped classroom teaching that takes place against the backdrop of MOOCs efficiently realizes the teaching with students as the major body and increases the learning efficiency of the students in the process.

## 3. CGA Model

This paper studies a combined model CNN-GRU-attention (CGA) for MOOC cheating detection. The model structure is shown in Figure 1.

It is proposed in this paper to use the Word2Vec function to encode the behaviors in the behavior sequence as dense real vectors, which are subsequently fed into the neural network model. The embedding layer serves as the model's input, and the real vector matrix is depicted in the following equation:

(1) $$\begin{array}{c} x_{1:n}=x_{1}⊕x_{2}⊕\cdots ⊕x_{n}. \end{array}$$

It is utilized as an input to the CNN layer, which performs convolution and pooling operations to extract the local spatial features in the behavior sequence after acquiring the vector-matrix representation of the behavior sequence. Additionally, it is used as an input to the GRU layer in order to extract the time series characteristics from the behavior sequence.

In this paper, 8 and 16 convolution kernels of sizes 3 and 5, respectively, are used to extract the local spatial information in the behavior sequence, and this operation can be represented by

(2) $$\begin{array}{c} c_{i}=f\left(\omega \cdot x_{1:i+h-1}+b\right), \end{array}$$

where *x*_1:*i*+*h*−1_ is subbehavior sequence vector matrix; then we can derive the feature map vector:

(3) $$\begin{array}{c} c=\left[c_{1},c_{2},\cdots ,c_{n-h+1}\right]. \end{array}$$

Then we perform the maximum pooling operation; the formula is as follows:

(4) $$\begin{array}{c} M_{i}=\max\left(c\right)=\max\left(c_{1},c_{2},\cdots ,c_{n-h+1}\right). \end{array}$$

Because pooling will cause the sequence structure to be disrupted, the pooled *M*_*i*_ is coupled into a feature vector *u*, as illustrated in the following equation:

(5) $$\begin{array}{c} u=\left(M_{1},M_{2}\cdots ,M_{K}\right), \end{array}$$

where *K* represents the number of cores.

Ordinary RNNs are capable of exploiting close-range semantic characteristics well, but they are plagued by the problem of vanishing gradients. There are several RNN versions that can be used to address this problem, including the LSTM and GRU. GRU is actually an enhancement of the LSTM algorithm. They are all based on the “gate mechanism,” which is used to memorize the previous sequence information in order to compensate for the inadequacies of conventional RNN. However, when compared to the three gate units of LSTM, GRU has only two gate units, namely the update gate and the reset gate, and its model is simpler, requiring fewer parameters and achieving a faster convergence speed than the LSTM.

The specific calculation process of GRU is as follows:

(6) $$\begin{array}{c} z_{t}=\sigma \left(\omega_{z}\cdot \left[h_{t-1},x_{t}\right]\right),\\ r_{t}=\sigma \left(\omega_{r}\cdot \left[h_{t-1},x_{t}\right]\right),\\ {\tilde{h}}_{t}=\tanh\left(\omega_{h}\cdot \left[r_{t}\times h_{t-1},x_{t}\right]\right),\\ h_{t}=\left(1-z_{t}\right)\times h_{t-1}+z_{t}\times {\tilde{h}}_{t},\\ {\overset{⟶}{h}}_{t}=GRU\left(x_{t},{\overset{⟶}{h}}_{t-1}\right),\\ {\overset{⟶}{h}}_{t}=GRU\left(x_{t},{\overset{\leftarrow }{h}}_{t-1}\right),\\ h_{t}=\left[{\overset{⟶}{h}}_{t},{\overset{\leftarrow }{h}}_{t}\right]. \end{array}$$

The flow chart of the GRU is shown in Figure 2.

As different weights are assigned to different input aspects of the model, the attention mechanism has the effect of increasing the influence of relevant information on the final outcome by allocating different weights to important information. The contribution of each behavior component to the final detection result varies depending on where you are in the process of detecting dishonest activity. This study presents the attention mechanism, which allows different weights to be assigned to different aspects on the basis of this information. Previously, the local feature vector and the time-series feature vector of the behavior sequence was produced by using CNN and GRU networks, respectively, to represent the behavior sequence. Because the local feature vector and the time series feature vector must be connected end-to-end in order to characterize the behavior sequence more completely, the new behavior sequence feature vector *z* is created, and it is then fed into the attention layer, where it is transformed into the final representation of cheating behavior.

The attention layer's computation process is illustrated in formulas (7)–(9), respectively

(7) $$\begin{array}{c} m_{i}=\tanh\left(\omega_{1}z_{i}+b\right), \end{array}$$

(8) $$\begin{array}{c} \alpha_{i}=\text{softmax}\left(\omega_{2}m_{i}\right), \end{array}$$

(9) $$\begin{array}{c} r=\sum_{i}\alpha_{i}z_{i}. \end{array}$$

## 4. Results and Observations

A total of 100 GB of desensitization data was obtained from the database of a MOOC online learning platform for this paper, which covered moreover 30,000 learners from September 2018 to September 2020. In order to learn behavioral trajectories, pick 75% of the samples as the training set and 25% of the samples as the validation set from the total number of samples.

Several approaches were chosen to conduct comparison tests on the validation set in order to evaluate the detection performance of the model presented in this research. The results are displayed in Figure 3 for CNN, LSTM, GRU, BiGRU, and CNN-GRU.

According to the experimental results, the CGA model suggested in this study has the maximum precision, recall, and AUC, with 96.67%, 97.32%, and 93.07%, respectively, according to the data. The first four sets of trials demonstrate that when compared to CNN and LSTM models, the GRU model performs significantly better in terms of cheating detection. The performance indicators of the model are enhanced when compared to the performance indicators of the unidirectional LSTM and GRU, showing that the bidirectional structure has been implemented. The BiGRU has the ability to extract additional contextual information from a sequence, which improves the ability to detect dishonest behavior during the sequence. The precision rate, recall rate, and AUC value of the detection model all improve dramatically after the attention mechanism based on GRU is implemented into the system. Significant traits have a greater impact on the classification of behavior sequences when they are given a higher weight. It is proposed in this research that the CGA network model integrates the advantages of network structures such as CNN, GRU, and attention mechanism and that the detection performance of the model is further enhanced.

According to Figure 4, we also analyzed the model inference time of different models. The longer the inference time, the more efficient and effective the algorithm performance.

Figure 5 depicts the AUC results obtained on the validation set following the application of LSTM. To train the training set before and after data augmentation, GRU, BiGRU, and the model in this paper were used, as was the model in this paper. The AUC of the CGA model proposed in this study is higher than that of other models, both before and after data augmentation, and is superior to other models.

## 5. Conclusion

MOOCs are a relatively advanced instructional modality that has a greater impact on the application. The ability to quickly and correctly detect the cheating behavior of MOOC English learners is critical for the further development of the MOOC platform and the provision of English education counseling. This paper has proposed a hybrid model CNN + GRU + attention for the detection of cheating in MOOC English. Furthermore, investigations have demonstrated the efficiency of the experimental procedure described in this study. The data amplification method is also employed in order to expand the sample size of minority categories, which is necessary due to the problem of unbalanced data categories in MOOC cheating behavior detection in real-world circumstances. Experiments have shown that model training following data amplification can help reduce the overfitting of the resulting model. It can be quite beneficial to the English education tutoring and instruction that is based on MOOCs in order to strengthen the generalization ability of the model [36].

## Figures and Tables

**Figure 1:** Structure of CGA.

**Figure 2:** Structure of GRU.

**Figure 3:** Comparison of different models.

**Figure 4:** Comparison of inference time.

**Figure 5:** Comparison of before and after data amplification.

## Data Availability

The data used to support the findings of this study are available from the corresponding author upon request.
